The article "Clinical Effect of Qili Qiangxin Capsule Combined with Sacubitril-Valsartan in Patients with Chronic Heart Failure" was retracted in 2023. Reasons: signs of a paper mill; suspected computer-generated content; unreliable results or conclusions; lack of ethics approval or compliance.

# Clinical Effect of Qili Qiangxin Capsule Combined with Sacubitril-Valsartan in Patients with Chronic Heart Failure

**DOI:** 10.1155/2022/8598806

**Published:** 2022-03-23

**Authors:** Jiafang Yao, Dan Liu

**Affiliations:** ^1^Department of Cardiology, The First People's Hospital, Affiliated to Huzhou Normal College, Huzhou 313000, China; ^2^Department of Nephrology, Central Hospital, Huzhou 313000, China

## Abstract

The clinical effect of Qili Qiangxin capsule combined with sacubitril-valsartan on patients with chronic heart failure was studied. We selected 108 patients with chronic heart failure in our hospital from March 2016 to January 2020 and divided them into a control group and a study group according to the random table method, with 54 cases in each. The control group took sacubitril and valsartan orally, and the study group took Qili Qiangxin pill on the basis of sacubitril and valsartan. The course of the treatment for 2 groups is 4 weeks. We compared the total effective rate of the treatment of the 2 groups for 4 weeks, cardiac function (left ventricular end-systolic volume (LVESV), left ventricular end-diastolic volume (LVEDV), and left ventricular ejection fraction (LVEF)) before and after 4 weeks of treatment, 6 min walking distance (6MWT), changes in cTnI and NT-proBNP levels, and adverse reactions. The total effective rate in the study group (90.74%) is higher than that in the control group (72.22%) (*P*＜0.05). After 4 weeks of treatment, the study group LVESV (45.23 ± 2.98 mm) and LVEDV (43.38 ± 4.01 mm) are lower than those of the control group ((49.98 ± 2.56 mm) and (50.75 ± 3.49 mm), respectively), while LVEF (47.38 ± 2.78%) is higher than that in the control group (42.08 ± 3.24%) (*P* ＜ 0.05). After 4 weeks of treatment, the study group 6MWT (476.58 ± 31.25 *m*) of patients with chronic heart failure is higher than that of the control group (396.52 ± 24.52 *m*) (P ＜0.05). After 4 weeks of treatment, the study group serum cTnI (0.36 ± 0.12 *μ*g/L) and NT-proBNP (276.91 ± 30.12 pg/ml) of patients with chronic heart failure are lower than those in the control group (0.87 ± 0.25 *μ*g/L) and (367.48 ± 48.57 pg/ml) (*P*＜0.05). There is no significant difference between the adverse reactions in the two groups (*P* ＞ 0.05). Conclusion: Xinbao pills combined with sacubitril and valsartan have a good effect on patients with chronic heart failure, which can improve the heart function and exercise endurance and reduce serum cTnI and NT-proBNP levels.

## 1. Introduction

Chronic heart failure refers to a series of clinical syndromes caused by chronic ventricular pressure and chronic primary diseases, which causes the decline of ventricular pump blood function, limb edema, pulmonary congestion, labor dyspnea, acute Qi, and fatigue [1–3]. In recent years, the prevalence of chronic heart failure has been continuously increased, seriously affecting people's quality of life [4]. At present, drugs are mainly used for patients with chronic heart failure [5]. In recent years, it has been found that patients with chronic heart failure can improve their treatment efficacy [6, 7]. Therefore, the purpose of this study is to explore the effect of Qili Qiangxin capsule and sacubitril-valsartan on the clinical effect of serum troponin I (cTnI) and N-terminal type B cerebral natriuretic peptide (NT-proBNP) levels in patients with chronic heart failure [8–12].

The rest of the paper is structured as follows. Methodology covering both data collection and data analysis is described in Section 2.  Section 3 presents the results of this research. This is followed by discussion which includes implications and limitations in Section 4. Lastly, we conclude this research and point out some potential future research directions in Section 5.

## 2. Data and Methods

### 2.1. General Information

A total of 108 patients with chronic heart failure from March 2016 to January 2020 are divided into control and study groups, 54 each, according to the randomized table method. The control group is 41 to 74 years (59.83 ± 7.58 years); 34 men and 20 women; course 2 to 12 years (7.98 ± 1.65 years); NYHA grade: 13 grade II, 27 grade III, and 14 grade IV. The study group is 43 to 75 years (60.34 ± 8.94 years); 32 males and 22 women; course 2 to 13 years (7.63 ± 1.80 years); NYHA grade: 11 II, 28 III, and 15 IV. The general data are not significantly different between the two groups (*P* ＞ 0.05).

Inclusion criteria are as follows: (1) diagnosis complies with the Chinese Guidelines for the Diagnosis and Treatment of Heart Failure 2014 Standard, (2) NYHA grades II ∼ IV, and (3) sign an informed consent form.

Exclusion criteria are as follows: (1) patients with acute heart failure and other cardiovascular system diseases, (2) patients with severe abnormal respiratory system and liver and kidney function, (3) allergic constitution, (4) patients with malignant tumors, and (5) patients with mental illness.

### 2.2. Method

The two groups are admitted to the hospital for basic treatment, including strong heart, diuresis, oxygen absorption, low-sodium diet, vasculogenic drugs, and treatment for basic diseases. Control group: oral sacubitril-valsartan (Beijing Novartis Pharmaceutical Co., Ltd.; specification: 0.1 g; J20190002) 100 mg/time, twice a day; study group: oral Qili Qiangxin capsule (Shijiazhuang Yiling Pharmaceutical Co., Ltd.; specification: 0.3 g; Z20040141) 4 grains/times, 3 times a day. Both group sessions are performed for 4 weeks.

### 2.3. Efficacy Criteria

1. Efficacy: NYHA cardiac function improved at level 2 or more for 4 weeks, and the main symptoms basically disappeared for 4 weeks;
2. Effective: NYHA improved at level 1 for 4 weeks, and the main symptoms improved for 4 weeks;
3. Invalid: NYHA for 4 weeks, and no main symptoms for 4 weeks.

### 2.4. Observation Indicators

1. Heart cardiac changes in two groups of patients with chronic heart failure: heart color Doppler ultrasound was used to examine the left ventricular end-systolic volume (LVESV), left ventricular end-diastolic volume (LVEDV), and left ventricular ejection fraction (LVEF);
2. Observation of the motor endurance changes in the two groups of chronic heart failure patients: 6 min walking test (6MWT) was used;
3. The serum cTnI and NT-proBNP levels are observed in the two groups of patients with chronic heart failure. The venous blood of 5 ml was collected before treatment and after 4 weeks of treatment. The supernatant was removed. Clear levels of cTnI and NT-proBNP were determined by an enzyme-linked immunosorbent assay;
4. Occurrence of adverse reactions in the two groups was observed.

The data were processed using the SPSS 25.0 software. The count data were analyzed using ^*2*^Inspection, and the measurement data were analyzed using *t*-test. *P* < 0.05 is considered as a statistically significant difference.

## 3. Results

### 3.1. Comparison of Efficacy between the Two Groups

The study group had 36 effective patients and 15 invalid patients The overall effectiveness in the study group of chronic heart failure patients (90.74%) is higher than that in the control group (72.22%) (*P* ＜ 0.05).  Table 1 shows the comparison of efficacy between the two groups of patients with chronic heart failure.

### 3.2. Comparison of Cardiac Function between the Two Groups

Both groups had lower LVESV and LVEDV than those before treatment, while LVEF is higher than that before treatment (*P* < 0.05); LVESV and LVEDV in the study group are lower than those in the control group, while LVEF in the study group is higher than that in the control group (*P* < 0.05).  Table 2 shows comparison of cardiac function between the two groups with chronic heart failure.

### 3.3. Comparison of 6MWT between the Two Groups

Both groups had higher 6MWT results in patients treated for 4 weeks than before treatment (*P* < 0.05); the study group had higher 6MWT in patients treated for 4 weeks than that of the control group (*P* < 0.05).  Table 3 displays 6MWT comparison between the two groups of patients with chronic heart failure.

### 3.4. Comparison of Serum cTnI and NT-proBNP Levels between the Two Groups

Serum levels of cTnI and NT-proBNP are lower in patients treated for 4 weeks than those before treatment (*P* < 0.05); the serum levels of cTnI and NT-proBNP in patients treated for 4 weeks are lower than those in the control group (*P* < 0.05).  Table 4 shows the comparison of serum cTnI and NT-proBNP levels between the two groups of patients with chronic heart failure.

### 3.5. Adverse Reactions

In the study group, 3 patients had gastrointestinal reaction, 2 patients were with fatigue, and one patient was with dizziness. In the control group, 2 patients had gastrointestinal reaction, 2 patients were with fatigue, and one patient was with dizziness. There is no significant difference in the adverse reactions between the two groups (P＞0.05).  Table 5 shows adverse reactions.

## 4. The Experimental Result Analysis

Chronic heart failure is mainly a very complex clinical disease caused by the accumulation of many heart classes. As a difficulty in cardiovascular disease, it has attracted wide attention by medical practitioners in recent years. Chronic heart failure is characterized by high incidence rate, high hospitalization rate, and high case fatality rate, which seriously threatens the life and health of patients. Therefore, adopting timely and effective methods to treat chronic heart failure are particularly important.

Sacubitril-valsartan tablets contain sacubitril and valsartan, in which sacubitril inhibits brain neprilysin, while valsartan inhibits angiotensin II, thus reducing aldosterone release, dilating blood vessels, improving urinary sodium excretion, and achieving therapeutic purposes. Qili Qiangxin capsule is mainly a Chinese patent medicine composed of *Astragalus*, ginseng, *Salvia miltiorrhiza*, accessory, Guizhi, Zetian, Ting Linzi, and tangerine peel, which has the effect of promoting water and eliminating swelling, promoting blood circulation and connecting collaterals, nourishing Qi and warming Yang. Modern pharmacological studies have shown that Qili Qiangxin capsule can inhibit the inflammatory response of the myocardial interstitium, reduce angiotensin II and aldosterone levels, improve vascular endothelial function, effectively inhibit the activation of the RASS system, effectively prevent ventricular remodeling, and improve myocardial function. In addition, Qili Qiangxin capsule is diuretic and improves the hemodynamic effect. This paper shows that the treatment in the study group of chronic heart failure patients are always more efficient than in the control group, It can be seen that the treatment with Qili Qiang heart capsule combined with sacubitril-valsartan in patients with chronic heart failure can improve the curative effect. LVESV and LVEDV in the study group with chronic heart failure treated for 4 weeks are lower than those in the control group and LVEF is higher than that in the control group. It can be seen that chronic heart failure patients are treated with sacubitril-valsartan to improve their heart function. The 6MWT of the study group of patients with chronic heart failure was higher than that in the control group. It is seen that patients with chronic heart failure treated with sacubitril-valsartan can improve exercise endurance.

## 5. Conclusion

Qili Qiangxin capsule combined with sacubitril-valsartan worked well in patients with chronic heart failure, improved cardiac function and motor endurance, and reduced serum cTnI and NT-proBNP levels. cTnI is a marker of myocardial injury, is a cardiomyocyte-specific antigen, and expressed almost in cardiomyocytes, while its levels rise significantly when myocardial damage occurs. BNP is mainly a diverse class of nerve hormones secreted by ventricular myocytes, whereas the ventricle oversecretes and releases BNP in pathological states such as ventricular wall pressure overload and abnormal volume expansion. Studies have reported that serum NT-proBNP level measurement has important value in judging the prognosis of heart failure, and the higher the level, the worse the patient heart function. This study showed that the serum levels of cTnI and NT-proBNP are lower in patients with 4 weeks of treatment than those in the control group, which showed that the use of Qili Qiangxin capsule with sacubitril-valsartan reduced the serum levels of cTnI and NT-proBNP in patients with chronic heart failure.

## Figures and Tables

**Table 1:** Comparison of efficacy between the two groups of patients with chronic heart failure.

Group	Example number	Excellence (%)	Valid (%)	Of no avail (%)	Total valid (%)
Study group	54	36 (66.67)	13 (24.07)	5 (9.26)	49 (90.74)
Control group	54	27 (50.00)	12 (22.22)	15 (27.78)	39 (72.22)
*χ* ^*2*^	—	—	—	—	6.136
*P* value	—	—	—	—	＜0.05

**Table 2:** Comparison of cardiac function between the two groups with chronic heart failure (±*s*).

Group	Example number	LVESV (mm)		LVEDV (mm)		LVEF (%)	
		Pretherapy	Treatment is performed for 4 weeks	Pretherapy	Treatment is performed for 4 weeks	Pretherapy	Treatment is performed for 4 weeks
Study group	54	56.23 ± 3.21	45.23 ± 2.98^*∗*^	60.81 ± 2.46	43.38 ± 4.01^*∗*^	37.28 ± 2.14	47.38 ± 2.78^*∗*^
Control group	54	55.47 ± 3.38	49.98 ± 2.56^*∗*^	60.47 ± 2.71	50.75 ± 3.49^*∗*^	36.98 ± 2.25	42.08 ± 3.24^*∗*^
*T*	—	1.198	8.885	0.683	10.188	0.710	9.123
*P* value	—	＞0.05	＜0.05	＞0.05	＜0.05	＞0.05	＜0.05

*∗P*＜0.05, compared with pretreatment.

**Table 3:** 6MWT comparison between the two groups of patients with chronic heart failure (±*s*, m).

Group	Example number	Pretherapy	Treatment is performed for 4 weeks
Study group	54	305.62 ± 26.21	476.58 ± 31.25^*∗*^
Control group	54	307.18 ± 29.98	396.52 ± 24.52^*∗*^
T	—	0.288	14.811
*P* value	—	＞0.05	＜0.05

^*∗*^ *P*＜0.05, compared with pretreatment.

**Table 4:** Comparison of serum cTnI and NT-proBNP levels between the two groups of patients with chronic heart failure (±*s*).

Group	Example number	cTnI (*μ*g/L)		NT-proBNP (pg/ml)	
		Pretherapy	Treatment is performed for 4 weeks	Pretherapy	Treatment is performed for 4 weeks
Study group	54	2.75 ± 0.43	0.36 ± 0.12^*∗*^	769.83 ± 64.23	276.91 ± 30.12^*∗*^
Control group	54	2.81 ± 0.65	0.87 ± 0.25^*∗*^	778.32 ± 85.96	367.48 ± 48.57^*∗*^
*T*	—	0.566	13.515	0.581	11.645
*P* value	—	＞0.05	＜0.05	＞0.05	＜0.05

^*∗*^ *P* ＜ 0.05, compared with pretreatment,

**Table 5:** Adverse reactions.

Group	Example number	Gastrointestinal reaction	Feeble	Dizzy	Incidence (%)
Study group	54	3	2	2	12.96
Control group	54	2	2	1	9.26
*χ* ^2^	—	—	—	—	0.375
*P* value	—	—	—	—	＞0.05

## Data Availability

The simulation experiment data used to support the findings of this study are available from the corresponding author upon request.
